The article "The cryoprotectant trehalose could inhibit ERS-induced apoptosis by activating autophagy in cryoprotected rat valves" was retracted in 2018. Reasons: false authorship; concerns about the data; concerns about the results or conclusions.

# The cryoprotectant trehalose could inhibit ERS-induced apoptosis by activating autophagy in cryoprotected rat valves

**DOI:** 10.1371/journal.pone.0194078

**Published:** 2018-03-09

**Authors:** Hongyan Wu, Qing Chang

**Affiliations:** Department of Cardiovascular Surgery, The Affiliated Hospital of Qingdao University, Qingdao University, Qingdao, China; Univerzitet u Beogradu, SERBIA

## Abstract

Valvular diseases are common health problems that are strongly related to high morbidity and mortality; aortic valve allograft transplantation may be a promising way to improve survival and relieve symptoms. However, ideal tissue viability has not been observed with common valve cryopreservation methods, which could lead to apoptosis and necrosis in cryopreserved tissue. It has been observed that trehalose plays a positive role by acting to maintain cell structures and protect cells from stress responses. In this study, we studied the effects of trehalose in protecting rat valve tissue from the cooling process. We found improved higher cell function in rat valves treated with trehalose during cryopreservation than in those treated with dimethyl sulphoxide (DMSO). To further explore the mechanisms, we found that trehalose could down-regulate the expression of cleaved caspase-3, an important molecule involved in cell apoptosis. In addition, treatment with trehalose also decreased Glucose-regulated protein 78 (GRP78) and CCAAT/enhancer-binding protein homologous protein (CHOP), the key proteins in the endoplasmic reticulum stress (ERS) process. Intriguingly, we observed that trehalose promotes cryoprotected rat valve cell autophagy via an mTOR-independent but p38 MAPK-dependent signaling pathway. Additionally, miR-221 and miR-32 have been implicated in such cell activities. In summary, our study offers a new and meaningful cryopreservation approach for valve allograft storage.

## Introduction

Congenital and acquired valvular diseases are worldwide problems with high morbidity and mortality. A wide range of common valvular diseases includes rheumatic heart disease, Takayasu arteritis, infective endocarditis and Marfan syndrome [1]. To date, there is nearly no effective medical treatment, though some surgical strategies, such as valve replacement, may improve survival and relief symptoms; these strategies started in the 1950s-1960s [2]. With the development of transplantation technology, cardiac centers decided to treat allografts with antibiotics and cryopreserve them at low temperature in order to prolong their life span [3]. However, these operations also obviously decrease allograft durability and activity and are likely related to some complicated stress process that compromises apoptosis, the endoplasmic reticulum or autophagy [4]. Therefore, finding effective cryopreservation methods for valve allografts is of remarkable interest.

The article "The cryoprotectant trehalose could inhibit ERS-induced apoptosis by activating autophagy in cryoprotected rat valves" was retracted in 2018. Reasons: false authorship; concerns about the data; concerns about the results or conclusions.

DMSO is a traditional agent in heart valve and vascular graft cryopreservation, and it is soluble in both aqueous and organic media [5]. Nevertheless, the application of DMSO also shows toxic effects that suppress allograft viability [6]. Additionally, some studies have reported that small carbohydrate sugars, such as trehalose and a-D-glucopyranosyl a-D-glucopyranoside, are verified to play a significant role in decreasing ice crystal formation and maintaining tissue proteins and membrane structures inside diverse types of cells [7].

Trehalose can be found in various organisms, including bacteria, yeast, fungi, invertebrates and plants, but is lacking in vertebrates. In some scientific and reliable studies, no dose-dependent adverse effects of trehalose were observed when it was added to the diet of humans at doses up to 10%. To further understand its positive properties, various research studies using different systems were started. For instance, Isachenko et al. found that adding trehalose to the preservation solution of a goat embryo could obviously up-regulate its viability [8]. Erdag et al. used trehalose and DMSO to preserve fetal skin; this method is better because it increases the quantity of skin cells compared with the glycerol and DMSO group [9]. In addition, trehalose has also been observed to have outstanding protectiveness in muscle, kidney and platelet cells [10–12].

Numerous studies have verified that trehalose has important biological properties, mainly exerted through the mTOR-independent signaling pathway. In the nervous system, Sovan Sarkar et al. found that trehalose could accelerate the clearance of mutant huntingtin by enhancing mTOR-independent autophagy [13–16]. Yuichi Honma et al. also observed that trehalose activated autophagy and decreased proteasome inhibitor-induced ERS and oxidative stress-mediated cytotoxicity in hepatocytes [17]. However, few reports have been published regarding the cryoprotective role of trehalose in valve allografts and the underlying mechanism.

In our previous studies, we found that trehalose could maintain the viability of rabbit aortic valve homografts in long-term storage, but further research is needed [18]. The aim of this study was to verify the mechanism of trehalose in protecting the valve transplant upon cryopreservation.

## Materials and methods

### 1. Materials

Eighty-eight male Wistar rats were sacrificed to obtain the aortic valves. Two aortic valves and their corresponding aortic wall (6 mm) and the myocardium under the valves (0.5 mm) were preserved. All animals were obtained from the Animal Institute of Affiliated Hospital of Qingdao University, and the studies we performed were conducted in the Animal Institute of Affiliated Hospital of Qingdao University according to the protocols approved by the Medical Experimental Animal Care Commission of Qingdao University.

The article "The cryoprotectant trehalose could inhibit ERS-induced apoptosis by activating autophagy in cryoprotected rat valves" was retracted in 2018. Reasons: false authorship; concerns about the data; concerns about the results or conclusions.

### 2. Cryopreservation

Nalgene® Mr. Frosty® Cryo 1°C Freezing Containers (No. 5100–0001, Thermo Fisher Scientific) were used to cryopreserve the samples. The samples were cryopreserved in liquid nitrogen for 4 and 16 weeks. The composition of the cryoprotectants in each group was as follows: control group, 10% DMSO, RPMI 1640, 10% fetal bovine serum, 100 U/L each penicillin and streptomycin; experimental group, 0–0.2 mol/L trehalose, RPMI 1640, 10% fetal bovine serum, 100 U/L each penicillin and streptomycin. In the p38 MAPK signaling pathway experiment, the control group was grown in 10% DMSO, RPMI 1640, 10% fetal bovine serum, and 100 U/L both penicillin and streptomycin, and the treatment group, 20 μmol/L SB203580 (p38 MAPK inhibitor, no. 5633; cell signaling technology), RPMI 1640, and 100 U/L 10% fetal bovine serum.

### 3. Determination of carbohydrate metabolism

Samples in each group were weighed and placed into RPMI-1640 nutrient solution containing 10% fetal bovine serum, and 2.5 mL of nutrient solution was needed for each 10 mg of tissue. Tissues were cultured at 37°C for 24 h. An automatic biochemical analyzer was used before and after culture to determine the glucose levels in the nutrient solution, and the difference between them was calculated.

### 4. Intracellular MDA measurement

Valve cellular extracts were prepared in ice-cold RIPA lysis buffer. Lysed cells were centrifuged at 13,000 g for 10 min to remove debris. The supernatant was subjected to the measurement of MDA (at 532 nm) levels with a microplate reader. MDA levels were then normalized to milligrams protein.

### 5. Western blot detection of apoptosis-related proteins

Total protein was extracted from samples with RIPA lysis buffer, separated by sodium dodecyl sulfate-polyacrylamide gel electrophoresis and transferred onto 0.45 μm PVDF membranes (Millipore). The following primary antibodies were used in the assays: antibodies for cleaved caspase-3 (no. 9654; Cell Signaling Technology, Danvers, MA, USA), GRP78 (no. 3183; Cell Signaling Technology), CHOP (no. 2895; Cell Signaling Technology), LC3A/B II/I (no. 12741; Cell Signaling Technology), p62 (no. 5114; Cell Signaling Technology), ATG-5 (no. 12994; Cell Signaling Technology), ATG-7 (no. 8558; Cell Signaling Technology), mTOR (no. 2983; Cell Signaling Technology), p-mTOR (Ser2448) (no. 5536; Cell Signaling Technology), p38 MAPK (no. 9212; Cell Signaling Technology), and p-p38 MAPK (no. 4511; Cell Signaling Technology), and β-actin (no. 3700; Cell Signaling Technology) was chosen as loading control.

The article "The cryoprotectant trehalose could inhibit ERS-induced apoptosis by activating autophagy in cryoprotected rat valves" was retracted in 2018. Reasons: false authorship; concerns about the data; concerns about the results or conclusions.

### 6. Quantitative reverse transcription-PCR (QRT-PCR)

Trizol (Invitrogen, Carlsbad, CA, USA) was used to extract the total RNA from tissues according to the instructions supplied by the manufacturer. Reverse transcription was conducted with Primescript RT Master Mix (Takara, Otsu, Japan), and cDNA was amplified using SYBR-Green Premix (Takara). U6 was used as a reference gene for miR-221 and miR-32, and the U6 forward primer was TCGCTTCGGCAGCACATA, and the U6 reverse primer was TTTGCGTGTCATCCTTGC. MicroRNA levels were detected using a Hairpin-itTM Quantitation PCR Kit (GenePharma, Shanghai, China). The data were analyzed by the delta Ct method. All PCR reactions were performed in duplicate.

### 7. Statistical analysis

Statistical analysis was carried out using the SPSS program (version 13.0; SPSS, Chicago, IL, USA). The statistical significance of differences between two groups was calculated by Student's t–test or χ2 test. Multiple comparisons were performed using a one-way ANOVA followed by Newman-Keuls test. Spearman's analysis was used in correlation analysis. P<0.05 was considered significant.

## Results

### 1. Trehalose performed better in cryopreservation of rat valves than DMSO

To determine whether trehalose is a better cryoprotectant in the cryopreservation of valves than DMSO, we first detected carbohydrate metabolism, which can indicate cell activity and MDA and can whether there is injury. Cryopreservation methods are shown above, and the concentrations of trehalose were 0, 0.05, 0.10, 0.15, and 0.20 mol/L. Samples cryopreserved for 4 and 16 weeks were chosen for each group. The results showed that there was no obvious cryopreservation difference in these groups at 4 weeks (Fig 1A and 1B). The group with 0.10 mol/L trehalose had the highest carbohydrate metabolism level (Fig 1C) and the lowest MDA level (Fig 1D) compared with other groups at 16 weeks. These results indicated that trehalose and DMSO had almost the same cryopreservation effect in short-time groups, while trehalose performed better in the long term with an optimum concentration of 0.1 mol/L. Thus, we selected 0.1 mol/L trehalose for our next studies.

**Fig 1:** Trehalose improved cell glucose consumption and decreased MDA content of cryopreserved valve cells. Valve cells were treated with DMSO or trehalose (0–0.20 mol/L). (A) Glucose consumption, valves were cryopreserved for 4 weeks. (B) MDA, valves were cryopreserved for 4 weeks. (C) Glucose consumption, valves were cryopreserved for 16 weeks. (D) MDA, valves were cryopreserved for 16 weeks. Data are expressed as the mean ± SD (*n* = 4 per group). *P < 0.05, **P < 0.01 versus the DMSO group.

The article "The cryoprotectant trehalose could inhibit ERS-induced apoptosis by activating autophagy in cryoprotected rat valves" was retracted in 2018. Reasons: false authorship; concerns about the data; concerns about the results or conclusions.

### 2. Trehalose could suppress apoptosis in cryoprotected rat valve cells via ERS signaling

To observe the mechanism of trehalose cryopreservation in rat valves, samples cryopreserved for 16 weeks were chosen from the trehalose 0.1 mol/L group and the DMSO group in order to extract protein and study apoptosis. The results showed that the cleaved caspase-3 level was lower in the trehalose group than in the DMSO group (Fig 2A and 2B). To further understand the mechanism by which trehalose inhibited valve cell apoptosis, we then detected important proteins in ERS signaling, such as CHOP and GRP78. The results showed that CHOP and GRP78 levels in the trehalose group were lower than those in the DMSO group (Fig 2C, 2D and 2E). These results indicated that trehalose might down-regulate apoptosis in cryoprotected valve cells via ERS signaling.

**Fig 2:** Effect of trehalose on apoptosis and ERS in cryopreserved valve cells. (A and B) Western blotting using a cleaved caspase-3 antibody on cryopreserved valve cells treated with trehalose (0.1 mol/L) or DMSO for 16 weeks. (C, D and E) Western blotting using GRP78 and CHOP antibodies on cryopreserved valves treated with trehalose (0.1 mol/L) for 16 weeks. Data are expressed as the mean ± SD (*n* = 20 per group). **P < 0.01, ***P < 0.001 versus the DMSO group.

### 3. Trehalose can inhibit ERS-induced apoptosis by activating autophagy in cryoprotected rat valve cells

To further study why trehalose inhibits ERS-induced apoptosis, we measured indicators of autophagy, such as LC3A/B-II/I, p62, ATG-5 and ATG-7, with a Western blot assay. The results showed that LC3A/B-II/I, ATG-5 and ATG-7 were up-regulated, while the p62 level was down-regulated in the trehalose group compared with that in the DMSO group (Fig 3). It is known that the activation of autophagy plays a significant role in the relief of ERS-induced apoptosis. These results verified that trehalose can inhibit ERS-induced apoptosis by activating autophagy in cryoprotected valves.

**Fig 3:** Effect of trehalose on autophagy in cryopreserved valve cells. (B, C, E and F) Western blotting using LC3A/B-II/I, p62, ATG-5 and ATG-7 antibodies on cryopreserved valve cells treated with trehalose (0.1 mol/L) or DMSO for 16 weeks. Data are expressed as the mean ± SD (*n* = 20 per group). **P < 0.01, ***P < 0.001 versus the DMSO group.

### 4. Trehalose activated autophagy through an mTOR- independent but p38 MAPK-dependent signaling pathway in cryoprotected rat valve cells

To determine whether or not trehalose activated autophagy through mTOR signaling in valve cells, key proteins in mTOR signaling, such as mTOR and p-mTOR (Ser2448), were measured by Western blot. The results showed that there was no significant difference in the level of p-mTOR (Ser2448) in the trehalose group compared with the DMSO group (Fig 4A and 4B), indicating the non-activation of mTOR signaling. Additionally, we also observed the protein level of p38 MAPK and p-p38 MAPK, which can usually regulate autophagy via an mTOR-independent pathway, and we found that the phosphorylation of p38 can be inhibited by trehalose (Fig 4C). Taken together, these results verified that trehalose activated autophagy through an mTOR-independent but p38 MAPK-dependent signaling pathway in cryoprotected rat valve cells.

The article "The cryoprotectant trehalose could inhibit ERS-induced apoptosis by activating autophagy in cryoprotected rat valves" was retracted in 2018. Reasons: false authorship; concerns about the data; concerns about the results or conclusions.

**Fig 4:** Trehalose activated the p38 MAPK signaling pathway in cryopreserved valve cells. (A, B and C) Western blotting using p-mTOR (Ser2448), mTOR, p38 MAPK and p-p38 MAPK antibodies on cryopreserved valve cells treated with trehalose (0.1 mol/L) or DMSO for 16 weeks. Data are expressed as the mean ± SD (*n* = 20 per group). ***P < 0.001 versus the DMSO group.

### 5. Trehalose might improve the effect of cryopreservation through miRNA in cryoprotected rat valve cells

To determine whether miRNAs might participate in the regulation of p38 MAPK signaling by trehalose, the levels of many miRNAs were measured by qRT-PCR in 20 pairs of samples from the trehalose 0.1 mol/L group and the DMSO group that were cryopreserved for 16 weeks. The results showed that miR-221 and miR-32, which were confirmed to regulate p38 MAPK signaling in prior reports, were decreased in the trehalose group compared with the levels in the DMSO group (Fig 5). Five pairs of samples that were used in the above protein analysis were also measured in the miRNA expression analysis that involved the 20 pairs. The correlation between cleaved caspase-3, LC3A/B II/I, p-p38 MAPK and miRNAs was analyzed. The results showed that miR-32 expression was significantly and positively correlated with cleaved caspase-3 levels, inversely correlated with LC3A/B II/I ratio and positively associated with p38 MAPK phosphorylation. Additionally, miR-221 expression was significantly and positively correlated with cleaved caspase-3 levels; no significant relevance was observed between miR-221 expression and LC3A/B II/I ratio or p38 MAPK phosphorylation. These results indicated that down-regulation of miR-32 may participate in trehalose-induced apoptosis inhibition, autophagy induction and p38 MAPK inactivation. miR-221 may participate in trehalose-induced apoptosis inhibition in cryoprotected rat valve cells. Thus, miR-32 and miR-221 can also act as biomarkers for assessment of the effect of cryopreservation on valves.

The article "The cryoprotectant trehalose could inhibit ERS-induced apoptosis by activating autophagy in cryoprotected rat valves" was retracted in 2018. Reasons: false authorship; concerns about the data; concerns about the results or conclusions.

**Fig 5:** Expression levels of miR-32 and miR-221 in cryopreserved valve cells. Twenty pairs of DMSO samples and trehalose samples were analyzed by qRT-PCR and normalized to U6 expression. (A and C) The bars represented relative miR-32 and miR-221 expression with the ratio of levels in DMSO samples to those in trehalose samples on a logarithmic scale. (B and D): miR-32 and miR-221 expression levels in DMSO samples and trehalose samples were compared with a paired Student’s t-test. *P < 0.05 versus DMSO group. (E, F and G): correlation analysis between miR-32 expression and cleaved caspase-3 level, LC3A/B II/I ratio and p38 MAPK phosphorylation. (H and J): correlation analysis between miR-221 expression and cleaved caspase-3 level, LC3A/B-II/I ratio and p38 MAPK phosphorylation. Spearman's analysis was used in the correlation analysis.

## Discussion

Cryopreservation is a promising way to maintain biological cell or tissue viability at low temperatures, such as below -80°C or even below –140°C; it has been proven to protect stored tissue materials effectively over the long term [19]. However, during the cryopreservation process, frozen tissue may have various severe responses as there are stress factors in the cooling environment, including cold stress, ice crystal formation inside or outside of cells, osmotic stress, and chemical toxicity from cryoprotectants, which could lead to morphological and functional damage and subsequent necrosis in cells [20–23]. Currently, DMSO is a common cryoprotectant that is used for freezing cells, tissues or other biological materials, but there are some reports that have observed its biological toxicity. Thus, finding new cryoprotectants to store cells safely and effectively is a significant contribution.

It has been noted that trehalose is the latest agent that can stabilize the cell membrane, protein and nucleic acid structure. In several studies, it has been proven that trehalose has unique anti-dehydration, anti-freezing, and anti-hypertonic protective effects [24, 25]. Because trehalose is a natural non-specific biological cryoprotectant, an increasing number of studies have focused on the cryopreservation use of trehalose. For example, Zhou Xinli used bovine serum and trehalose as a platelet extracellular protective agent that greatly increased platelet extracellular survival [26]; Jia Xiaoming and others have shown that for protection of the skin *in vitro*, trehalose was significantly better than DMSO [27]; and the research of Campbell LH shows that the protective effect in organs of the combined use of the impermeable cryoprotective agent trehalose and the protective agent DMSO on permeability at low temperature was significantly better than that of a single agent [28]. To take a step toward understanding the mechanism of action of trehalose, various studies on cell reactions were undertaken.

The article "The cryoprotectant trehalose could inhibit ERS-induced apoptosis by activating autophagy in cryoprotected rat valves" was retracted in 2018. Reasons: false authorship; concerns about the data; concerns about the results or conclusions.

In this study, we found that trehalose had the same cryopreservation effect as DMSO at 4 weeks, but with an increased storage period, trehalose performed better than DMSO. A higher carbohydrate metabolism level with glucose consumption showed that trehalose could keep valve cells active, while a lower MDA level suggested that trehalose could protect the valve cells from low-temperature injury. More importantly, we first found that trehalose was promising as a better cryoprotectant than DMSO in valve cryopreservation; this coincided with other studies on trehalose in other organs. We also determined that the optimum concentration for trehalose in cryopreservation was 0.1 mol/L.

Considering the emerging data, we speculated that trehalose might up-regulate valve cell viability through the inhibition of apoptosis. Intriguingly, the results showed that after cryopreservation and thawing, a decreased expression level of cleaved caspase-3 was detected in rat valve cells treated with trehalose compared to the levels in the DMSO group. It has been previously reported that severe ERS could result in apoptosis [29], and in normal cells, it could result in endoplasmic reticulum (ER) biosynthesis, folding and transporting proteins. If stress factors such as cold, starvation, or ischemia occurred, the balanced environment in cells would breakdown, and unfolded or misfolded proteins might accumulate in the ER, leading to ERS [30]. We found that trehalose down-regulated GRP78 and CHOP proteins compared with the DMSO group, suggesting that this agent could inhibit ERS in cryoprotected rat valve cells. It is known that the activation of autophagy plays a significant role in the relief of ERS-induced apoptosis in damaged organelles; misfolded proteins in the cell can be degraded to maintain cell and body homeostasis. We suggest that trehalose may inhibit ERS-induced apoptosis by activating autophagy in cryoprotected valves. To confirm this idea, we determined whether autophagy was involved in the effects of trehalose; we selected LC3A/B-II/I and p62 as our target proteins. In cell autophagy, the conversion of LC3A/B-I to LC3A/B-II is an important process for autophagosome maturation, enabling lysosome fusion and autophagosome cargo degradation [31]. The protein p62 is a selective substrate for autophagy [32]. We observed that trehalose could up-regulate the ratio of LC3A/B-II/I, ATG-5 and ATG-7 and down-regulate the protein level of p62, demonstrating that this agent could activate autophagy to inhibit ERS-induced apoptosis. Then, our study thoroughly focused on the mechanism of trehalose in the cryopreservation of rat valves, a topic that had never been studied. Some studies have discussed the functions and mechanisms of trehalose on cells and proved that trehalose could induce autophagy, depending on mTOR [33, 34]. Within an mTOR-independent modulation of autophagy, some cellular mechanisms, including cAMP/Epac/Ins [35], inositol [36], Ca^2+^/calpain [37], c-Jun N terminal kinase (JNK)/Beclin1/PI3K [38], and p38/Atg [39], have been discovered. In this study, we found that trehalose could activate autophagy through an mTOR-independent but p38 MAPK-dependent signaling pathway in cryoprotected rat valve cells.

The article "The cryoprotectant trehalose could inhibit ERS-induced apoptosis by activating autophagy in cryoprotected rat valves" was retracted in 2018. Reasons: false authorship; concerns about the data; concerns about the results or conclusions.

Interestingly, we found that miR-221 and miR-32, which were confirmed to regulate p38 MAPK signaling in past reports, were down-regulated in the trehalose group compared to those in the DMSO group. We think that down-regulation of miR-221 and/or miR-32 might participate in trehalose-induced apoptosis inhibition, autophagy induction and p38 MAPK inactivation in cryoprotected rat valve cells. However, the mechanism by which trehalose down-regulates miR-221 and miR-32 is not clear and needs further investigation. Finally, we drew the conclusion that trehalose performed better than DMSO in the cryopreservation of rat valves with an optimum concentration of 0.1 mol/L. Trehalose could inhibit ERS-induced apoptosis by activating autophagy via an mTOR-independent but p38 MAPK-dependent signaling in cryoprotected rat valve cells.

## Conclusions

Supplementation with trehalose resulted in higher glucose consumption activity and less MDA content. Trehalose was able to protect valve cells from apoptosis induced by the cooling process and may be recommended to suppress the induction of ERS and promote the autophagy process via an mTOR-independent but p38 MAPK-dependent signaling pathway. Additionally, miR-221 and miR-32 might participate in this reaction; these mechanisms need further studies.

## Supporting information

S1 Fig P38 MAPK inhibitor suppressed autophagy in cryopreserved valve cells. (DOCX)
